# Comparative Anesthesia Effect of Brachial Plexus Block Based on Smart Electronic Medical Ultrasound-Guided Positioning and Traditional Anatomical Positioning

**DOI:** 10.1155/2021/6676610

**Published:** 2021-02-25

**Authors:** Zhaoxiang Yu, Yang Liu, Chunlei Zhu

**Affiliations:** ^1^Department of Anesthesiology, Affiliated Hospital of Beihua University, Jilin 132012, Jilin, China; ^2^Department of Endocrine, Affiliated Hospital of Beihua University, Jilin 132012, Jilin, China; ^3^Department of Hand and Foot Surgery, Affiliated Hospital of Beihua University, Jilin 132012, Jilin, China

## Abstract

With the intensification of population aging, the improvement of visualization technology, and the concept of accelerated rehabilitation surgery, the anesthesia method of upper extremity surgery is gradually changing. However, these methods are often caused by anatomical variations and often have low block success rates and patient satisfaction. The neuroanatomical position should be accurately located so that the puncture needle is right next to the nerve bundle or in the nerve sheath. This is very important for implementing accurate brachial plexus anesthesia. This article uses ultrasound-guided positioning technology and traditional anatomical positioning technology for brachial plexus block treatment, aiming to explore the anesthesia effect of brachial plexus block with different techniques. This article selects 120 patients undergoing brachial plexus block surgery for forearm or hand surgery and divides these 120 patients into 6 groups with 20 people in each group. The first 3 groups were treated with brachial plexus block using ultrasound-guided positioning technology. The latter 3 groups were treated with brachial plexus block using traditional anatomical positioning technology. Experiments proved that during anesthesia, compared with the ultrasound group, the heart rate of the traditional anatomy group was significantly decreased (*P* < 0.05), and the average arterial pressure of the six groups of patients at each time point had no statistical difference (*P* > 0.05). This shows that whether it is ultrasound-guided positioning technology or traditional anatomical positioning technology, it has no effect on the average arterial pressure of the patient at each time point. In addition to intuitive and accurate viewing of needle and nerve contact, ultrasound real-time guidance allows intuitive viewing of anesthesia. This is a special advantage of nerve block under ultrasound guidance.

## 1. Introduction

In recent years, brachial plexus block has played an important role in clinic, especially in orthopedic shoulder, upper limb, and hand surgery. Compared with general anesthesia, brachial plexus block anesthesia has simple operation, less physiological interference, and fewer complications, and is safe, economical, and effective. In recent years, nerve stimulants and ultrasound positioning technology have been gradually introduced into clinical practice to make nerve block technology more advanced, and the application of network block anesthesia has become more and more common [1]. Commonly used lattice arm pathways include axillary approach, intramuscular sulcus approach, subclavian approach, and subclavian paravascular approach. In traditional axillary brachial plexus block, the methods of locating anatomical landmarks and acupuncture to find abnormal feelings are often used. After the puncture is in place, a certain volume of local anesthetic is injected to complete the nerve block. Axillary brachial plexus insufficiency is clinically more clinical. Typically, the radial nerve travels deep into the axillary artery due to nerve anatomy. Therefore, if the axillary brachial plexus nerve is blocked, the use of only local anesthetics will cause the upper extremity radial block to be incomplete, affecting the blocking effect. Local anesthetics have little effect on resolving imperfect blocks.

There have been many research results in foreign brachial plexus block methods. The nerve stimulator can stimulate the peripheral nerves by sending out stimulating currents, thereby causing the corresponding innervation muscle activities. It is the first commonly used nerve location to implement anesthesia method. However, it is still a blind puncture location, and the current repeatedly stimulates the nerve, which brings great discomfort to the patient. Sambataro proposed the application of doppler ultrasound blood flow monitor to identify the subclavian artery and for the first time performed an ultrasound-guided supraclavicular brachial plexus block [2]. Assi C et al. also found that the enhanced echo needle can significantly improve the visibility of deep vein catheterization, shorten the puncture time, improve the puncture success rate, and reduce the risk of puncture-related complications [3, 4]. Lian proposed adding a small dose of fentanyl to local anesthetics for brachial plexus block, which significantly improved the success rate of the block, shortened the onset time, prolonged the sensory block time, and had no obvious side effects [5].

In recent years, there have been more and more studies on brachial plexus block in China. With the improvement of science and medical technology, the research on brachial plexus block has become more and more mature, but the results of the research are still not as good as foreign countries. Among them, the ultrasound-guided nerve block has been widely used clinically because it can intuitively display the needle route of the puncture needle, the position of the needle tip, and the dynamics of local anesthetic diffusion. Harminder et al. proposed that the placement of the puncture position requires a high degree of patient cooperation. For those patients who do not cooperate well due to injuries or other reasons, they often cause inaccurate positioning or difficult puncture, and the blocking effect is often unsatisfactory [6]. Bonaretti et al. proposed that abnormal sensations or muscle movements cannot be explored one by one. Different degrees of nerve insufficiency are more common and affect the effect of anesthesia [7]. Insufficiency of nerves is one of the urgent problems to be solved in nerve block technology [8]. Brogden et al. proposed a finite element model of needle puncture viscoelasticity and simulated the interaction of needle and soft tissue in MATLAB for uniform and nonuniform soft tissue materials [9].

In brachial plexus block, when large doses or high concentrations of ropivacaine are used, the motor and sensory nerves tend to be completely blocked, but it may cause local anesthetic toxicity or postoperative discomfort due to nerve paralysis. At the same time, it will affect the surgeon's evaluation of postoperative motor nerve function recovery, especially for soft tissue surgery that may cause nerve damage. This article presents ultrasound-guided positioning and traditional anatomical positioning techniques to explore different anesthesia techniques by comparing drug onset time, analgesic retention time, blocking effect, motor function recovery time, and impact on the myocardium using the same treatment method. This effect provides a reference material for clinical application.

## 2. Anesthesia Effect of Brachial Plexus Block with Intelligent Electronic Medical Ultrasound-Guided Positioning and Traditional Anatomical Positioning

### 2.1. Medical Ultrasound-Guided Positioning and Tracking Technology

#### 2.1.1. Ultrasonic Positioning Guidance Technology

The common ultrasonic wave in clinical medicine is applied to the piezoelectric crystal on the ultrasonic probe by a high-frequency alternating current signal. The transducer has an inverse piezoelectric effect; that is, electrical energy generates mechanical energy, and its surface will produce high-frequency compression and expansion. Drive the surrounding medium to vibrate together, so ultrasonic waves are generated [10, 11]. Ultrasound imaging is widely used because of its many advantages, but speckle gives ultrasound images its unique granular appearance. As an inherent image attribute in the field of synthetic aperture radar imaging, ultrasound imaging, and laser, there have been two types for a long time [12]. The opposite understanding is that the speckle texture observed by the naked eye does not correspond to the underlying tissue structure, which reduces the clarity and quality of the image, and increases the difficulty of the doctor's diagnosis. So blotches are noise in the image and need to be suppressed and removed. In clinical medicine, it is difficult to determine the position of the needle axis and the tip of the puncture needle due to the influence of noise such as artifacts aiming at the 2D ultrasound imaging problem of ultrasound-guided puncture surgery.

#### 2.1.2. Ultrasound Image Preprocessing

The main purpose of image preprocessing is to suppress the influence of image speckles on ultrasound images, improve the quality of ultrasound images during the ultrasound-guided needle puncture process, that is, speckle noise, and reduce the ultrasonic imaging system's ability to distinguish between puncture needles and soft tissues, affecting the diagnosis of doctors during percutaneous puncture surgery [13].

*(1). Wavelet Transform*. Ultrasound image has high requirements for edge detail and is a nonstationary signal, so the traditional Fourier transform-based signal denoising method can no longer meet the requirements [14, 15]. Ultrasonic speckle suppression and noise removal methods can be largely divided into spatial domain local statistical filtering, anisotropic diffusion filtering, and wavelet transform-based filtering.

Since the filtering denoising effect based on wavelet transform is better than Kuan filtering, SRAD filtering, Gamma/MAP filtering, Wiener filtering, enhanced frost filtering, Lee filtering, and other standard speckle removal techniques on ultrasound images [16], the wavelet transform-based filter transformation to remove speckles in ultrasound images is used. The speckle noise model can be expressed as follows:

(1) $$\begin{array}{c} g\left(x,y\right)=f\left(x,y\right)h\left(x,y\right)+\eta \left(x,y\right). \end{array}$$

In the formula, *x* and *y*, respectively, represent the rows and columns in the image, *f*(*x*, *y*) is the image that is not contaminated by other noises and needs to be restored, *η*(*x*, *y*) is the image additive noise, *h*(*x*, *y*) is the image multiplicative noise, and *g*(*x*, *y*) is the actual acquisition noisy image to be processed. The damage of the multiplication noise to the original information of the image is much larger than that of the additive noise, and the effect of additive noise on the ultrasound image is relatively small, so it is generally neglected. Therefore, formula (1) can be rewritten as

(2) $$\begin{array}{c} g\left(x,y\right)=f\left(x,y\right)h\left(x,y\right). \end{array}$$

In order to separate the speckle noise from the original signal, through logarithmic transformation, the speckle multiplicative noise is transformed into speckle additive noise. Formula (2) is rewritten as

(3) $$\begin{array}{c} \mathrm{lg}g\left(x,y\right)=\mathrm{lg}f\left(x,y\right)+\mathrm{lg}h\left(x,y\right). \end{array}$$

Then, use wavelet discrete transform to degrade the ultrasonic image with speckle noise.

*(2). Wavelet Threshold Denoising*. The wavelet domain threshold denoising algorithm can select wavelet denoising thresholds on different scales and then use this threshold to directly or indirectly process the wavelet transform coefficients, especially the wavelet coefficients corresponding to noise, in order to achieve the purpose of denoising or suppressing noise [17, 18]. The function of the wavelet threshold function is to remove the wavelet transform coefficients with small values and keep or shrink the wavelet transform coefficients with large values. From this, we can see that it is very important to choose the appropriate wavelet domain value function and wavelet denoising threshold. Hard threshold function:

(4) $$\begin{array}{c} W_{w}=\left\{\begin{array}{cc} X_{w}, & \text{where}\left|W_{w}\right|\geq T,\\ 0, & \left|W_{w}\right|<T. \end{array}\right. \end{array}$$

Semi-soft threshold function:

(5) $$\begin{array}{c} W_{w}=\left\{\begin{array}{cc} \text{sign}\left\{X_{w}\right\}\left(\left|X_{w}\right|-a\cdot T\right), & \left|X_{w}\right|\geq T,\\ 0, & \left|X_{w}\right|<T. \end{array}\right. \end{array}$$

Soft threshold processing function:

(6) $$\begin{array}{c} W_{w}=\left\{\begin{array}{cc} \text{sign}\left\{X_{w}\right\}\left(\left|X_{w}\right|-T\right), & \left|X_{w}\right|\geq T,\\ 0, & \left|X_{w}\right|<T, \end{array}\right. \end{array}$$

where *W*_*w*_ is the wavelet transform coefficient after soft thresholding, *X*_*w*_ is the original wavelet coefficient, *T* is the threshold, and *a* ∈ (0,1) is the coefficient.

*(3). Selection Threshold*. The maximum communication delay that the user can tolerate under the cloud and fog architecture is guaranteed, and the user's request is processed within the acceptable communication delay. Another key to the wavelet domain threshold denoising method is to choose an appropriate threshold size. The general threshold expression is

(7) $$\begin{array}{c} T=\chi_{n}\sqrt{2\;\log\left(M\times N\right)}. \end{array}$$

Among them, *χ*_*n*_ is the noise standard value, and *M* × *N* is the row and column of the image.

(8) $$\begin{array}{c} T=\frac{\beta \partial^{2}}{\partial_{y}}. \end{array}$$

Among them, *β* is the subband scale parameter, which determines the decomposition level and the size of the subband; ∂ is the noise standard deviation; ∂_*y*_ is the standard deviation within the subband.

(9) $$\begin{array}{c} R\left(T\right)=\sum_{i=1}^{N}{\left(\left|y_{i}\wedge T\right|\right)}^{2}+\sigma_{n}^{2}-\frac{2\sigma_{n}^{2}}{N}\sum_{i=1}^{N}I\left(\left|y_{i}\right|<T\right). \end{array}$$

Among them, ∧ is the smaller value between two numbers. The threshold can be easily obtained after the function is minimized in the above formula, and its value is

(10) $$\begin{array}{c} T^{*}=\arg\min R\left(T\right),\;T>0. \end{array}$$

The BayesShrink criterion can better select the effective threshold for the ultrasound image containing speckle noise. The signal and noise meet:

(11) $$\begin{array}{c} T=\frac{{\hat{\sigma }}_{n}^{2}}{{\hat{\sigma }}_{x}},\\ {\hat{\sigma }}_{n}=\frac{\text{median }\left(\left\{\left|W_{k}\right|\in HH_{1}\right\}\right)}{0.6745},\\ {\hat{\sigma }}_{x}=\sqrt{\max\;\left({\hat{\sigma }}_{y}^{2}-{\hat{\sigma }}_{n}^{2},0\right)}. \end{array}$$

Among them, ${\hat{\sigma }}_{x}$ is the estimated standard deviation of the subband coefficients, ${\hat{\sigma }}_{n}^{2}$ is the noise estimation variance, and *HH*_1_ is the diagonal detail subband after multiscale wavelet decomposition.

(12) $$\begin{array}{c} {\hat{\sigma }}_{y}^{2}=\frac{1}{N}\sum_{k=1}^{N_{f}}W_{k}^{2}. \end{array}$$

Among them, *N*_*j*_ is the number of coefficients *W*_*k*_ in the *j* subband, and ${\hat{\sigma }}_{y}^{2}$ is the estimated variance of the original image observation value.

#### 2.1.3. Binary Image

After wavelet threshold denoising, the binarization of puncture needle ultrasound images during needle puncture needs to go through three steps of smoothing, thresholding, and morphological processing [19, 20]. Use MLESAC algorithm to calculate. The model of the points in the ultrasound image can be expressed as

(13) $$\begin{array}{c} p\;\left(e|M\right)=\gamma \;{\left(\frac{1}{\sqrt{2\pi }\sigma }\right)}^{d}\exp\;\left(-\frac{e^{2}}{2\sigma^{2}}\right)+\left(1-\gamma \right)\frac{1}{v}, \end{array}$$

where *γ* is the mixing coefficient and *v* is the diameter or size of the error search box of the mixed model. Randomly select two data points in the ultrasound binary image as the base *d* of the ultrasound positioning *M* model, use the selected two points as the minimum sampling set for parameter estimation, and obtain the negative logarithm of the cost function [21, 22]. The maximum consensus set is the maximum estimate $\hat{M}$ of the puncture needle model *M*:

(14) $$\begin{array}{c} \text{Loss}\left(e\right)=-\log\;p\left(e|M\right),\\ \hat{M}=\underset{M}{\arg\min}\left\{\sum_{i=1}^{n}\text{Loss}\left(e|M\right)\right\}. \end{array}$$

When the algorithm is initialized, the mixing coefficients *γ*=0.5 , *η*_*i*_ are the indicator variables of the *i* sampling, where *η*_*i*_=1 represents the interior point and *η*_*i*_=0 represents the exterior point. The expectation maximization algorithm is used to calculate the *γ* of the *i* sample:

(15) $$\begin{array}{c} \gamma =\frac{1}{n}\sum_{i=1}^{n}P\left(\eta_{i}=1|\gamma \right)=\frac{1}{n}\sum_{i=1}^{n}\frac{P_{i}}{P_{i}+P_{o}},\\ p_{ix}=\gamma \;{\left(\frac{1}{\sqrt{2\pi }\sigma }\right)}^{d}\exp\;\left(-\frac{e^{2}}{2\sigma^{2}}\right),\\ p_{o}=\left(1-\gamma \right)\frac{1}{v}. \end{array}$$

Among them, *p*_*i*_ is the inner point probability of a certain sampling, *p*_*o*_ is the outer point probability of a certain sampling, and *n* is the total sampling times. The position of the needle shaft can be estimated through the iteration of the algorithm [23, 24].

### 2.2. Anesthesia Effect of Brachial Plexus Block

#### 2.2.1. Safety and Application of Intravenous Local Anesthesia

The safety and effectiveness of anesthesia are the basic principles of clinical anesthesia. As an ancient regional anesthesia method, intravenous local anesthesia is an ideal method of anesthesia especially for short surgical operations on the upper extremities. With the development of anesthesia technology, it has been extended to the fields of pain and postoperative recovery treatment. Under the recommended dosage and administration speed, intravenous anesthesia injection of lidocaine can take effect quickly, and the risk is extremely low [25, 26]. When performing intravenous local anesthesia, a tourniquet should be tied to the limb. Tourniquets can help maintain local anesthesia in the distal blood vessel. When the tourniquet is released, the analgesic effect immediately disappears. Therefore, postoperative pain relief cannot be guaranteed, and joint use of other pain medications, that is, multidimensional pain medications, is required.

#### 2.2.2. Ultrasound Positioning

Brachial plexus injury is the most complicated peripheral nerve injury, especially open injury, which is difficult to treat and is a difficult clinical problem. Therefore, it is particularly important to understand the blood vessels and anatomical structures of the brachial plexus. After general anesthesia, the effect of local anesthesia is good [27, 28]. Scan the nerve area with the ultrasound probe to image the lower axis of the nerve. The piercing needle is inserted on the side of the longitudinal axis of the catheter and enters the tissue in the direction of the ultrasound beam. Follow the guidance of the ultrasound visualization to orient the puncture needle to reach the nerve block. Local anesthetics are injected when the needle approaches the nerve and penetrates the ultrasound fiber sheath around the nerve.

#### 2.2.3. Nerve Block

The analgesic effect provided by respiratory anesthesia is not good. In surgery, this method combined with respiratory anesthesia can provide the most effective analgesia. Brachial plexus block in the forelimbs has a series of complications, including intravascular injections, intrapleural injections, and nerve damage. The use of ultrasound guidance is to reduce the occurrence of complications [29, 30]. Under ultrasound guidance, the nerves block the brachial plexus, thereby paralyzing the forelimbs at the distal end of the elbow joint, which has a strong application effect for the operation of the distal elbow joint. This method can play a nerve block effect in the operation of the distal end of the elbow joint, and the effect is significant in all local nerve block methods.

#### 2.2.4. Anesthesia Monitoring and Indicators

All anesthetics are dangerous, and the most important way to ensure the safety of anesthesia is careful monitoring. Anesthesia should be a completely reversible process. To make anesthesia reversible, monitoring of a variety of physiological indicators is required. Under certain drugs or nerve stimulation, the heart rate will increase [31, 32]. The increase in heart rate can reflect the degree of response of the animal body to pain, and it will respond more quickly than other pain. The evaporation of the opening during the operation, the evaporation of body fluids during the laparotomy, the preoperative water and fasting, pain response, the use of painkillers and sedatives, abdominal washing operations, etc. will increase or decrease the animal's body temperature. The changes in body temperature within a certain range are controllable [33, 34].

#### 2.2.5. Clinical Significance of Local Anesthesia

Prioritizing the management of pain during surgery is not only an ethical consideration, but also to reduce the adverse effects of acute pain during surgery and reduce postoperative mortality. Intravenous local anesthesia is widely used in human medicine, but there is no corresponding model for research. More statistics are conducted through clinical patient experiments, which has certain risks [35, 36]. Establishing intravenous anesthesia experiments on animals and understanding the changes in dosage and methods on experimental animals will help to establish animal models of intravenous local anesthesia. Ultrasound-guided lower brachial plexus block is a more advanced clinical analgesic method, which can improve the effectiveness of clinical anesthesia analgesia.

## 3. Experimental Design of Anesthesia Effect of Brachial Plexus Block

### 3.1. Test Subject

The objects of this experimental study are 120 patients who were hospitalized in *X* Hospital from January 18 to December 2020, and 120 patients with forearm or hand surgery under brachial plexus block, ASA I-II, male and female, age 18 to 60 years, weighing 49 to 83 kg. The 120 patients were divided into 6 groups with 20 people in each group. The first 3 groups were treated with brachial plexus block using ultrasound-guided positioning technology, and the latter 3 groups were treated with brachial plexus block using traditional anatomical positioning technology. The experiment was approved by the hospital ethics committee, and all patients understood and signed an informed consent form for anesthesia.

### 3.2. Experimental Method

#### 3.2.1. Preparation before Anesthesia

All patients were injected intramuscularly with 10 mg of diazepam and 0.5 mg of atropine 30 minutes before surgery. After entering the room, an intravenous channel was created and an appropriate amount of sodium lactate Ringer's solution was provided for fluid replenishment, in addition to routine noninvasive blood pressure monitoring, electrocardiogram, pulse oximetry, and respiratory rate monitoring, and oxygen mask (5 L/min). The anesthesia assistant prepared the blocker and, when ready, began anesthesia.

#### 3.2.2. Anesthesia Implementation

Brachial plexus block anesthesia was performed with a nerve stimulator-assisted two-point approach of the inferior axillary approach. Routinely disinfect the skin and spread a hole towel. First touch the pulse of the axillary artery at the axillary, and then move along the artery, up to the point where the pulse of the axillary artery at the lower edge of the pectoralis major muscle disappears, slightly downward, and take the highest point of the artery pulse as the puncture point. Look for the median nerve, mark the flexion reflex of the wrist to the radial side, the flexion reflex of the index and middle fingers, and the downward stimulation of the palm. The injection method is the same as the above, and 8 ml of local anesthetic is injected. The radial nerve is found inside the axillary artery, which is marked by the stimulating movement of the wrist or finger extension, and the ulnar nerve is marked by the stimulating movement of the wrist to the ulnar flexion reflex, the little finger and index finger flexion reflex, and the adduction of the thumb. According to the above injection method, each inject 8 ml of local anesthetic, a total of 32 ml.

#### 3.2.3. Intraoperative Maintenance

If insufficiency occurs, inject an intraoperative local injection of 1% lidocaine 5–10 ml, or intravenously add fentanyl 0.1 mg to maintain the operation. If the block is ineffective, change to general anesthesia, and the experiment excludes cases of transition to general anesthesia. Intraoperative heart rate <50 bpm, intravenous infusion of atropine 0.25 mg.

### 3.3. Observation Index

Observe and record the patients' mean arterial pressure and heart rate before anesthesia, 5 minutes after injection, at the beginning of the operation, 30 minutes during the operation, and after the operation. Record the time of anesthesia operation (the time from the beginning of the puncture to the completion of the catheterization), the onset time of the block (the time after the injection of the drug until the pain begins to decrease), the anesthesia effect, and record the postoperative 0.5, 1, 2, 4, 8, and 12 hVAS score and sedation effect score, record the intraoperative and postoperative analgesic use of the two groups of patients and the number of PCA compressions within 48 hours after the operation, and record the intraoperative and postoperative complications.

### 3.4. Statistical Data Processing Method

SPSS23.0 software was used for data processing, and the count data was expressed in percentage (%), *k* is the number of data in this experiment, *σ*^2^ is the variance of all survey results, and *P* < 0.05 indicates that the difference is statistically significant. The formula for calculating reliability is shown in

(16) $$\begin{array}{c} a=\frac{k}{k-1}\left(1-\frac{\sum \sigma_{i}^{2}}{\sigma^{2}}\right). \end{array}$$

## 4. Anesthesia Effect of Brachial Plexus Block

### 4.1. Index Reliability Test and Patient Condition

#### 4.1.1. Evaluation Index System Based on Index Reliability Testing

Reliability refers to the stability and reliability of the questionnaire. This article adopts the *α* coefficient method created by L. J. Cronbach. The *α* coefficient can be obtained by Reliability Analysis in SPSS software. It is generally believed that the *α* coefficient above 0.8 indicates that the effect of index setting is very good, and above 0.7 is also acceptable. Here, we analyze the reliability of each type of object, and the reliability index we choose for each type of object is slightly different. The results are shown in Table 1. In the experimental stage, our experimental object is the artistic visual form of ceramic murals and the data source is the questionnaire that was issued and retrieved. Here, we publish questionnaires by age group to reduce significant differences.

It can be seen from Figure 1 that the data obtained from various indicators such as drug onset time, analgesic maintenance time, blocking effect, motor function recovery time, and impact on the myo cardium have an acceptable impact on this experiment (*α* > 0.7); the anesthesia effect of brachial plexus block with ultrasound-guided positioning and traditional anatomical positioning can be analyzed from the side.

#### 4.1.2. Comparative Analysis of Patients

Table 2 shows the comparison of age, gender, height, weight, anesthesia operation time, operation time, and intraoperative blood loss of each group of patients.

There was no significant difference in age, gender, height, weight, anesthesia operation time, operation time, and intraoperative blood loss in each group, *P* > 0.05. The specific situation is shown in Figure 2.

### 4.2. During Anesthesia, Blood Circulation, Breathing Rate, Ramsay Sedation Score, and Motor Block

#### 4.2.1. Hemodynamic Parameters during Anesthesia

Here, we performed ultrasound-guided positioning and traditional anatomical positioning for brachial plexus block therapy on the patients and recorded hemodynamic parameters during anesthesia (using Guangdong Baolight A8 multifunction monitor for noninvasive monitoring), and the blood flow of six groups of patients at each time point (kinetic parameters) is shown in Tables 3 and 4.

During anesthesia, compared with the ultrasound group, the heart rate of the traditional anatomy group decreased significantly (*P* < 0.05), and the average arterial pressure at each time point of the six groups had no statistical difference (*P* > 0.05). This shows that neither ultrasound-guided positioning techniques nor traditional anatomical positioning techniques always affect the patient's mean arterial pressure. However, since conventional anatomical positioning techniques require traumatic positioning and anesthesia of the brachial plexus nerve, blood input and output can be unstable. The heart rate dropped significantly, as shown in Figure 3.

#### 4.2.2. Respiratory System Parameters during Anesthesia

Here, we performed ultrasound-guided positioning and traditional anatomical positioning for brachial plexus block treatment and recorded respiratory system parameters during anesthesia (using Guangdong Baolight A8 multifunction monitor for noninvasive monitoring). The respiratory system parameters of the six groups of patients at each moment are shown in Tables 5 and 6.

During the period of anesthesia, there was no statistical difference in blood oxygen saturation of the six groups of patients at each time point (*P* > 0.05), and there was no statistical difference in the respiratory rate of the six groups of patients at each time point (*P* > 0.05). This shows that neither the ultrasound-guided positioning technology nor the traditional anatomical positioning technology has any effect on the patient's blood oxygen saturation and respiratory rate at all times. The specific situation is shown in Figure 4.

#### 4.2.3. Ramsay Sedation Score and Motor Block during Anesthesia

Here, we performed ultrasound-guided positioning and traditional anatomical positioning for brachial plexus block therapy and recorded Ramsay sedation scores during anesthesia. The Ramsay sedation scores of the six groups of patients at each time point are shown in Table 7.

During anesthesia, the Ramsay sedation score of the ultrasound group was significantly higher than that of the traditional anatomy group (*P* < 0.05), and the score of the traditional anatomy group was significantly higher at 24 h (*P* < 0.05). The specific situation is shown in Figure 5.

Here, we performed ultrasound-guided positioning and traditional anatomical positioning for brachial plexus block therapy on the patient and recorded the motor block time and motor recovery time during anesthesia. The results are shown in Table 8.

It can be seen from Figure 6 that there was no statistical difference in the onset and recovery time of exercise block in each group (*P* > 0.05). The specific situation is shown in Figure 6.

### 4.3. VAS Analgesia Score at Each Time Point after Operation

Here, we performed ultrasound-guided positioning and traditional anatomical positioning for brachial plexus block treatment and recorded postoperative VAS analgesia scores of 0.5, 1, 2, 4, 8, and 12 hours. The VAS analgesia scores of the six groups of patients at each time point are shown in Table 9.

Compared with the traditional anatomy group, the VAS score of the ultrasound group increased significantly at 2–12 h after surgery (*P* < 0.05), while the traditional anatomy group only slowly increased after 2 h (*P* < 0.05). This shows that the ultrasound guidance technology can pinpoint nerves accurately and monitor them in real time, increase nerve block success rate, and reduce complications caused by puncture, takes less time, and is more effective. The specific situation is shown in Figure 7.

## 5. Conclusions

In clinical anesthesia, the anesthesiologist needs to choose the approach of brachial plexus block and local anesthetics according to the conditions of the hospital, the patient's surgical method and the familiarity with ultrasound, etc., and ultimately provide the patient with a good upper limb surgical anesthesia effect and postoperative analgesia effect. Compared with general anesthesia, when real-time ultrasound-guided regional nerve block anesthesia is proficient, brachial plexus block can greatly reduce the block operation time and the onset time of sensory and motor block and reduce the incidence of related complications. These advantages reduce the number of hospital stays, save medical resources, promote rapid postoperative recovery of patients, speed up the turnover rate of hospital patients, improve the efficiency of medical workers, and improve the satisfaction of patients and surgeons.

With the development of visualization, ultrasound guidance technology can accurately find nerves, monitor them in real time, increase nerve block success rate, reduce complications caused by puncture, take less time, and apply effects quickly. Ultrasound guidance technology has been widely used in anesthesia and is an area of continuous development. The speckle is considered a noise signal in the ultrasound image, and the BayesShrink criterion wavelet soft threshold technique is used to remove the speckle in the ultrasound image. After Otsu threshold and morphological processing, the needle is finally punctured based on the MLESAC algorithm, and the image is processed to obtain the position of the puncture needle in the 2D ultrasound image. BIS monitoring can more accurately and objectively monitor a patient's intraoperative pain and sedation and more accurately reflect a patient's intraoperative sedation. In future research, more advanced scientific monitoring techniques should be gradually introduced to make the research more complete.

The ideal regional block anesthesia should have the characteristics of fast onset, long duration, strong analgesia, and fewer complications. When ultrasound is applied to brachial plexus block, it can improve the accuracy of the block and reduce the occurrence of related complications. The real-time guidance of ultrasound has the advantages of reducing the dose of anesthesia without reducing the success rate and prolonging the duration of the block and the duration of analgesia. At the same time, it can reduce the risk of local anesthetic toxicity. In addition to the needle-nerve contact that can be seen intuitively and accurately, the ultrasound real-time guidance can also intuitively see the diffusion path of anesthetic drugs. This is a special advantage of nerve block under ultrasound guidance. Nerve injury is a common complication of traditional peripheral nerve block anesthesia. Due to the introduction of ultrasound technology, the risk of nerve damage during block anesthesia is gradually reduced. It is mainly related to the avoidance of intranerve injection under ultrasound guidance.

## Figures and Tables

**Figure 1:** Indicator reliability test analysis chart.

**Figure 2:** Comparison and analysis of patient conditions.

**Figure 3:** Analysis chart of mean arterial pressure at each moment during anesthesia.

**Figure 4:** Analysis of blood oxygen saturation at each moment during anesthesia.

**Figure 5:** Ramsay sedation score analysis diagram at each moment during anesthesia.

**Figure 6:** Analysis diagram of motor block during anesthesia.

**Figure 7:** VAS score analysis diagram at various times after operation.

**Table 1:** Data sheet of evaluation index system for index reliability testing.

	Very clear and convenient	Clear and convenient	General	Not clear enough	Chaotic	Cronbach alpha
Drug onset time	0.317	0.398	0.164	0.083	0.038	0.9133
Analgesia maintenance time	0.111	0.201	0.323	0.199	0.166	0.8196
Blocking effect	0.184	0.284	0.249	0.187	0.096	0.8362
Exercise function recovery time	0.112	0.176	0.352	0.204	0.156	0.7819
Effect on myocardium	0.067	0.110	0.398	0.258	0.167	0.7432

**Table 2:** Patient condition comparison data sheet.

Group		Age	Gender (men/women)	Height	Weight	Anesthesia operation time	Operation time	Intraoperative blood loss
Ultrasound group	A	47.32	15/5	170.25	71.91	23.95	72.75	5.75
	B	43.26	14/6	169.10	68.05	25.10	72.00	4.50
	C	38.64	14/6	169.95	63.27	24.30	69.00	2.75
Anatomy group	D	46.12	13/7	169.25	69.14	25.45	77.25	10.85
	E	43.10	13/7	177.32	70.47	23.50	83.25	8.45
	F	38.89	14/6	165.29	64.18	23.10	68.25	8.00
P		0.935	0.964	0.977	0.936	0.952	0.972	0.933

**Table 3:** Data table of average heart rate at each moment during anesthesia.

Group		8 h	12 h	24 h	36 h	48 h
Ultrasound group	A	76.45	77.55	80.90	80.55	80.22
	B	77.29	77.37	80.39	80.57	80.32
	C	79.17	77.69	81.37	81.26	80.75
Anatomy group	D	80.12	78.84	75.70	75.50	74.97
	E	75.55	75.60	71.19	72.70	74.30
	F	76.33	73.12	71.66	72.94	71.32
P		0.008	0.004	0.002	0.001	0.001

**Table 4:** Average arterial pressure data table at each moment during anesthesia.

Group		8 h	12 h	24 h	36 h	48 h
Ultrasound group	A	91.50	92.95	92.10	91.25	90.65
	B	92.95	92.50	90.25	91.95	91.45
	C	94.55	92.75	92.65	90.20	90.33
Anatomy group	D	92.66	91.52	87.80	88.80	88.40
	E	93.12	91.45	90.25	89.42	88.36
	F	93.69	91.83	89.36	89.13	88.79
P		0.219	0.174	0.236	0.197	0.183

**Table 5:** Data sheet of blood oxygen saturation at each moment during anesthesia.

Group		8 h	12 h	24 h	36 h	48 h
Ultrasound group	A	100.16	100.24	100.27	100.39	100.56
	B	99.77	99.96	99.96	100.24	100.47
	C	100.00	100.27	100.42	100.57	100.70
Anatomy group	D	100.08	100.08	100.06	99.55	99.27
	E	99.68	99.51	99.87	100.09	100.16
	F	98.32	98.76	98.97	99.28	98.76
P		0.109	0.164	0.133	0.129	0.107

**Table 6:** Respiratory rate data table at each moment during anesthesia.

Group		8 h	12 h	24 h	36 h	48 h
Ultrasound group	A	19.09	18.54	18.42	18.03	17.89
	B	18.65	18.35	18.43	17.98	17.73
	C	18.65	18.65	18.42	18.42	18.32
Anatomy group	D	18.77	18.69	18.42	18.42	18.23
	E	19.54	19.27	19.03	18.89	19.14
	F	18.14	18.41	18.47	18.55	18.29
P		0.197	0.209	0.183	0.168	0.227

**Table 7:** Ramsay sedation score data sheet at each moment during anesthesia.

Group		8 h	12 h	24 h	36 h	48 h
Ultrasound group	A	1.77	1.52	1.61	2.22	2.49
	B	1.77	1.69	2.65	2.41	2.17
	C	1.84	1.77	2.36	2.12	1.59
Anatomy group	D	1.69	1.61	3.84	3.46	3.17
	E	1.63	1.56	3.11	2.67	1.87
	F	1.59	1.52	3.27	3.19	2.97
P		0.001	0.001	0.001	0.001	0.001

**Table 8:** Data sheet of motor block during anesthesia.

Group		Onset time of motor block	Exercise recovery time
Ultrasound group	A	11.706	246.79
	B	11.304	252.66
	C	10.904	256.50
Anatomy group	D	10.401	261.87
	E	10.137	265.33
	F	10.026	259.87
P		0.197	0.216

**Table 9:** VAS score data sheet at various times after operation.

Group		0.5 h	1 h	2 h	4 h	8 h	12 h
Ultrasound group	A	0	0.70	3.07	8.17	8.26	7.56
	B	0	0.69	1.97	6.11	6.45	6.14
	C	0	0.62	1.78	5.47	5.32	5.19
Anatomy group	D	0	0	0	2.24	4.08	4.52
	E	0	0	0	1.72	3.50	4.00
	F	0	0	0	3.32	3.98	5.72
P		0.010	0.008	0.008	0.004	0.002	0.001

## Data Availability

No data were used to support this study.

## References

[1] Zhou M., Wang Y., Liu Y., Tian Z. (2019). An information-theoretic view of WLAN localization error bound in GPS-denied environment. *Institute of Electrical and Electronics Engineers Transactions on Vehicular Technology*.

[2] Sambataro S., Cervino G., Fiorillo L., Cicciù M. (2018). Upper first premolar positioning evaluation for the stability of the dental occlusion. *Journal of Craniofacial Surgery*.

[3] Assi C., Kheir N., Samaha C. (2017). Optimizing patellar positioning during total knee arthroplasty: an anatomical and clinical study. *International Orthopaedics*.

[4] Zhao J., Huang J., Xiang Y. (2021). Effect of a protective coating on the surface integrity of a microchannel produced by microultrasonic machining. *Journal of Manufacturing Processes*.

[5] Zhou L., Zhu H., Shi D. (2019). Transverse facial cleft (macrostomia) repair: modification of a traditional technique. *Journal of Plastic, Reconstructive & Aesthetic Surgery: JPRAS*.

[6] Harminder S., Vogel R. W., Lober R. M. (2016). Intraoperative neurophysiological monitoring for endoscopic endonasal approaches to the skull base: a technical guide. *Scientifica*.

[7] Bonaretti S., Vilayphiou N., Chan C. M. (2017). Operator variability in scan positioning is a major component of HR-pQCT precision error and is reduced by standardized training. *Osteoporosis International*.

[8] Chen C.-H., Song∗ F., Hwang F.-J., Wu L. (2020). A probability density function generator based on neural networks. *Physica A: Statistical Mechanics and Its Applications*.

[9] Brogden C. M., Armstrong R., Page R., Milner D., Norris D., Greig M. (2018). Use of triaxial accelerometry during the dance aerobic fitness test: considerations for unit positioning and implications for injury risk and performance. *Journal of Dance Medicine & Science*.

[10] Soto Iglesias D., Duchateau N., Kostantyn Butakov C. B. (2017). Quantitative analysis of electro-anatomical maps: application to an experimental model of left bundle branch block/cardiac resynchronization therapy. *Institute of Electrical and Electronics Engineers Journal of Translational Engineering in Health and Medicine*.

[11] Ichiko T., Igarashi C., Sugisaki M., Wakae-Morita S., Ito H., Kobayashi K. (2016). A study on head positioning during panoramic radiography of the pterygopalatine fossa. *Shika Hoshasen*.

[12] Shankar K., Elhoseny M., Lakshmanaprabu S. K. (2020). Optimal feature level fusion based ANFIS classifier for brain MRI image classification. *Concurrency and Computation: Practice and Experience*.

[13] Haugen T., Buchheit M. (2016). Sprint running performance monitoring: methodological and practical considerations. *Sports Medicine*.

[14] Attard S., Couto J. G., Mackay S. (2016). Anatomical site markers (ASMs): evaluation of their use among Maltese radiographers. *Journal of Medical Imaging and Radiation Sciences*.

[15] Song H., Brandt-Pearce M. (2012). A 2-D discrete-time model of physical impairments in wavelength-division multiplexing systems. *Journal of Lightwave Technology*.

[16] Elhoseny M., Shankar K. (2019). Optimal bilateral filter and convolutional neural network based denoising method of medical image measurements. *Measurement*.

[17] Graham-Paulson T. S., Perret C., Watson P., Goosey-Tolfrey V. L. (2016). Improvement of sprint performance in wheelchair sportsmen with caffeine supplementation. *International Journal of Sports Physiology and Performance*.

[18] Keller E. J., Semaan E., Lee J. (2016). The direct and indirect costs of ultrasound-guided peripherally inserted central catheter repositioning at a large academic medical center. *Journal of the Association for Vascular Access*.

[19] Woolgar M. (2016). Ultrasound-guided positioning of transpyloric feeding tubes in critically ill infants. *Sonography*.

[20] Takeshita J., Inata Y., Ito Y. (2020). Dynamic needle tip positioning for ultrasound-guided placement of a peripherally inserted central catheter in pediatric patients. *Journal of Cardiothoracic and Vascular Anesthesia*.

[21] Cajozzo M., Palumbo V. D., Mannino V. (2018). Ultrasound-guided port-a-cath positioning with the new one-shoot technique: thoracic complications. *La Clinica Terapeutica*.

[22] Li M., Ballhausen H., Hegemann N.-S. (2017). Comparison of prostate positioning guided by three-dimensional transperineal ultrasound and cone beam CT. *Strahlentherapie Und Onkologie*.

[23] Torres Macho J., García Sánchez F. J., Garmilla Ezquerra P. (2018). Positioning document on incorporating point-of-care ultrasound in Internal Medicine departments. *Revista Clínica Española (English Edition)*.

[24] Midha D., Mandal A. K., Kumar A. (2017). Ultrasound guidance for central venous catheterization: a step further to prevent malposition of central venous catheter before radiographic confirmation. *Indian Journal of Critical Care Medicine*.

[25] Li J. W., Songthamwat B., Samy W., Blanch X. S., Karmakar M. K. (2017). Ultrasound-guided costoclavicular brachial plexus block sonoanatomy, technique, and block dynamics. *Regional Anesthesia and Pain Medicine*.

[26] Amini R., Kartchner J. Z., Nagdev A., Adhikari S. (2016). Ultrasound-guided nerve blocks in emergency medicine practice. *Journal of Ultrasound in Medicine*.

[27] Ward F., Faratro R, McQuillan R. F (2017). Ultrasound-guided cannulation of the hemodialysis arteriovenous access. *Seminars in Dialysis*.

[28] Fang G., Wan L., Mei W., Yu H. H., Luo A. L. (2016). The minimum effective concentration (MEC90) of ropivacaine for ultrasound-guided supraclavicular brachial plexus block. *Anaesthesia*.

[29] Shrestha G. S., Shrestha M., Shrestha B. (2020). Ultrasound guided central venous cannulation in ICU: retrospective analysis of a single center experience. *Journal of Advances in Internal Medicine*.

[30] Winwood P. W., Posthumus L. R., Cronin J. B., Keogh J. W. L. (2016). The acute potentiating effects of heavy sled pulls on sprint performance. *Journal of Strength and Conditioning Research*.

[31] Melton M. S., Monroe H. E., Qi W., Lewis S. L., Nielsen K. C., Klein S. M. (2017). Effect of interscalene brachial plexus block on the pulmonary function of obese patients: a prospective, observational cohort study. *Anesthesia & Analgesia*.

[32] Noguchi S., Kitayama M., Saito J., Nakai K., Hirota K. (2018). Rebound pain occurring after a single-shot brachial plexus block: two case reports. *The Journal of Japan Society for Clinical Anesthesia*.

[33] Paluvadi V., Manne V. S. K. (2017). Effect of addition of fentanyl to xylocaine hydrochloride in brachial plexus block by supraclavicular approach. *Anesthesia: Essays and Researches*.

[34] Sakae T. M., Marchioro P., Schuelter-Trevisol F., Trevisol D. J. (2017). Dexamethasone as a ropivacaine adjuvant for ultrasound-guided interscalene brachial plexus block: a randomized, double-blinded clinical trial. *Journal of Clinical Anesthesia*.

[35] Rastogi B., Arora A., Gupta K. (2016). Effect of midazolam and 0.5% levobupivacaine combination in ultrasound-guided supraclavicular brachial plexus block for upper limb surgeries-a clinical study. *Open Anesthesiology Journal*.

[36] Yang L. L., Ji J. S., Zhao Z. W. (2016). Effect comparison of ultrasound-guided lower extremity nerve block and spinal anesthesia in ankle surgery. *Zhonghua Yi Xue Za Zhi*.

